# DNAPred_Prot: Identification of DNA-Binding Proteins Using Composition- and Position-Based Features

**DOI:** 10.1155/2022/5483115

**Published:** 2022-04-13

**Authors:** Omar Barukab, Yaser Daanial Khan, Sher Afzal Khan, Kuo-Chen Chou

**Affiliations:** ^1^Department of Information Technology, Faculty of Computing and Information Technology in Rabigh, King Abdulaziz University, P. O. Box 344, Rabigh, 21911 Jeddah, Saudi Arabia; ^2^Department of Computer Science, School of Systems and Technology, University of Management and Technology, P.O. Box 10033, C-II, Johar Town, Lahore 54770, Pakistan; ^3^Department of Computer Sciences, Abdul Wali Khan University Mardan, Pakistan; ^4^Gordon Life Science Institute, Boston, MA 02478, USA

## Abstract

In the domain of genome annotation, the identification of DNA-binding protein is one of the crucial challenges. DNA is considered a blueprint for the cell. It contained all necessary information for building and maintaining the trait of an organism. It is DNA, which makes a living thing, a living thing. Protein interaction with DNA performs an essential role in regulating DNA functions such as DNA repair, transcription, and regulation. Identification of these proteins is a crucial task for understanding the regulation of genes. Several methods have been developed to identify the binding sites of DNA and protein depending upon the structures and sequences, but they were costly and time-consuming. Therefore, we propose a methodology named “DNAPred_Prot”, which uses various position and frequency-dependent features from protein sequences for efficient and effective prediction of DNA-binding proteins. Using testing techniques like 10-fold cross-validation and jackknife testing an accuracy of 94.95% and 95.11% was yielded, respectively. The results of SVM and ANN were also compared with those of a random forest classifier. The robustness of the proposed model was evaluated by using the independent dataset PDB186, and an accuracy of 91.47% was achieved by it. From these results, it can be predicted that the suggested methodology performs better than other extant methods for the identification of DNA-binding proteins.

## 1. Introduction

DNA (Deoxyribonucleic acid) is a blueprint for the cell. It contains information that is encoded for all our characteristics. A living thing's DNA is what makes a living thing a living thing. It is an essential part of reproduction that is transmitted from parents to offspring. There are four primary functions of DNA, commonly known as replication, encoding information, gene expression, and mutation and recombination. But DNA does not do this all alone; thousands of proteins in the cells help DNA to regulate DNA functions. Actions related to DNA are carried out with the help of specific proteins in living cells. These actions are carried out as the result of protein-DNA synergy [1]. Non-specific or specific binding between DNA and protein is involved in achieving regulation. Proteins that attach to DNA for such governance are known as DNA-binding proteins. These DNA-binding proteins contain a domain of DNA-binding and have an affinity for single- as well as double-stranded DNA. At different stages of life, these functional proteins play a vital role [2].

Moreover, DNA-protein binding plays an imperative role in the gene study and the development of a living body. Their research also helps in an inspection of the human body. It helps in the identification of the procedure of actions taking place in the body such as ailment, growth, development, changes, and improvement.

In the development of cell and growth systems, an important role is played by the transcription factor. It usually resides in a cell with an inactive state, and the existence of ligand TF becomes active. Desireless activation is responsible for many diseases such as inflammation, development disorder, autoimmunity, cancer, and abnormal hormone responses. Therefore, keeping a continuous record of DNA-binding proteins is of significant interest. It helps in the identification of, and treatment of diseases such as abnormal TF activity, cancers and genetic disorder which includes haemophilia, colour blindness, and many more. DNA-BP also plays an integral part in prokaryotic host defence in the shape of restriction enzymes. Binding of DNA with protein is shown in Figure 1.

Many experimental approaches used in biology have been adopted for the identification of DNA-binding proteins. These include X-ray crystallography [3], chromatin immunoprecipitation with DNA microarrays [4], and filter-binding assays [5]. These methods enable us to make exact identification of DNA-protein binding, but these mechanisms for proteins structures recognition are laborious, time-consuming, and require comprehensive material and expanse.

There are two practical approaches for the identification of sequences based on protein behaviour. One is the ML algorithms, to make improvements and expert model with derived numeral feature vector and query sequence forecasting. The second is the elicitation of organic information enclosed in the sequence of the protein and its metamorphosis into a comparable numeral vector of the features. Modern computational approaches for the identification of DNA binding protein are classified into two main classes: (1) Machine learning-based and (2) template-based.

Based on machine learning, DNA-binding protein prediction methodologies are divided into two general categories: structure-based [8, 9] and sequence-based [10–14] prediction. Higher identification rates can be achieved by the structure-based prediction of DNA-binding protein. Still, due to the inadequacy of sufficient knowledge about the structure of a protein, these approaches are not used on a large scale for the perception of high-throughput sequences. For predicting the function of a protein, new approaches are based on sequences of amino acids. By the result of bountiful experiments and methods, it realizes that proteins or primary polypeptide structure resembles the structural arrangement of polypeptide after wrapping and their methods are also very identical [15]. Template-based methods are also known as a template-based methodology because this identifies the consequential correspondence of protein sequences or structure among a known template and a query to bind DNA, to determine and evaluate the DNA-binding priority of sequences that are targeted [16, 17]. In contrary to the template-based approach, machine learning methodology determines a similar forecasting model to predict by analyzing and identifying the arrangement and pattern in feature space input. Some cases are support vector machine (SVM) [11, 12, 18–20], random forest [21], neural network [22–25], nearest neighbors' algorithm [23], naïve Bayes classifier [26, 27], and ensemble classifiers [28–30]. The process of identifying DNA binding protein by utilizing machine learning techniques requires two essential steps: (1) compatible feature extraction and (2) selection of suitable classification algorithm. The extant predictive methodology can be divided into two sections based on feature elicitation methods: (1) from protein structure extract appropriate features [31–34] and (2) relevant feature extraction from amino acid sequences [8, 35–38]. For DNA-binding protein recognition, more accurate and authentic results can be obtained using a structure-based prophecy technique [39]. Still, for this, a 3D structure with a high resolution of the protein sequence is required.

Thus, until now, for the identification of DNA-binding protein, many computing techniques direct from their amino acid sequences have been proposed and suggested. These approaches independently analyze and probe four distinct kinds of a feature of protein sequences and ciphering sequences [11, 39–42]. Categorically, the four specific types consist of (1) structural information, (2) functional and compositional information, (3) information about evolution, and (4) physicochemical properties. The four distinct categories of encoding procedures are as follows: (i) OCTD (global strategy) overall composition-transition-distribution, (ii) SSA transformation (local procedure) called split amino acid, (iii) ACC transformation (nonlocal approach) autocross covariance, and (iv) position-specific scoring matrix distant transformation known as “PSSM-DT”. These procedures have been considered deep in their related scrutinize work [28, 39, 43, 44].

There exist few recent studies which perform prediction of DNA-binding proteins using multiple features and machine learning classifiers. In 2022, Zhang et al. proposed a novel method for prediction of DNA-binding proteins by using features from amino acid composition and evolutionary information of protein sequences. Later, these features were fed to an XGboost classifier [45]. Furthermore, Harini et al. in 2022 created a database named ProNAB for DNA and protein complexes [46]. Jia et al., in 2021, proposed KKDBP, a classifier for the prediction of DNA-binding proteins using multiple PSSM feature fusions and random forest as a classifier [47]. In 2021, Hu et al. proposed TargetDBP+, which performed prediction of DNA-binding proteins using five convolutional features and SVM classifier [48]. Qian et al. in 2021, extracted six sequence-based features and used Multiple Kernel Learning-based on Centered Kernel Alignment for fusion of these features. Further, SVM was used for the classification of DNA-binding proteins [49]. Zou et al. proposed FTWSVM-SR, which used multiple sequence-based features and SVM as a classifier for predicting DNA-binding proteins [50]. Zou et al. also proposed MK-FSVM-SVDD, another predictor for DNA-binding protein prediction using six features with central kernel alignment and SVM as classifier [51]. However, the accuracy of all these proposed methods still has room for improvement. Nevertheless, most of the suggested approaches are inadequate in their capability to describe protein-DNA binding. Therefore, it is vital to develop a new strategy for the prediction of DNA-binding proteins accurately and efficiently and to compare it with existing state-of-the-art techniques.

The present work focuses on the identification of DNA-binding proteins through sequences. There are usually two goals for predicting DNA-binding proteins with different techniques: (1) to help scientists for the development and get covet data and (2) to encourage academic studies for appropriate fields. For establishing a sound analytical protein identification system, we need to deal with following the 5-step rule that includes (a) a valid standard dataset, (b) sample formulation, (c) algorithm for operation purpose, (d) performing cross-validation, and (e) friendly user web server for forecasting which is publicly accessible. The proposed system is highly accurate as compared to the previously existing methods and is easy to opt for as it only uses sequence-based features of proteins to identify them as DNA binding or non-DNA binding.

## 2. Materials and Methodology

The methodology is divided into five steps, the first aspect, which is “A valid benchmark,” is discourse here in this section. The protein sequence benchmark dataset was obtained from UniProtKB. At first, all types of sequences are passed out from a process of CD-HIT, which stands for Cluster Database at High Identity with Tolerance, and is initially composed by Weizhong Li and is now available publicly. The basic functionality of CD-HIT is to take input in FASTA format and remove similar or highly similar sequences from the dataset. The purpose is to reduce the size of the dataset by removing redundant or highly matching sequences from the dataset. So, for a benchmark dataset used in this study, sequences' identity cut-off is set to 60%. Redundant sequences or 60% identical were removed out, and a dataset is formed. All sequences of the obtained dataset are classified into two categories: (a) positive and (b) negative. These sequences of the DNA-binding protein are available in the dataset named “Dataset”. The dataset contains 57,194 DNA-binding protein sequences in which there are positive 11,526 sequences. Moreover, to check the robustness of the proposed methodology model, an independent dataset PDB 186 [40] has also been used. There are 93 binding proteins and 93 nonbinding protein sequences in an independent dataset. The performance of the proposed method has been compared with state-of-the-art methodologies. The details of datasets are shown in Table 1.

For the identification of DNA-binding protein, the methodology followed includes data collection from UniProt, applying preprocessing and filtration techniques, after that calculating the features obtained, in the end, training the classifier and getting the results, as shown in Figure 2.

### 2.1. Extracting Features

The second step describes how the dataset samples are devised into proper expressions of mathematics which equate and compare these samplings with aimed biological class in a remarkably precise, efficient, and accurate way.

Such a formulation of samples is essential depending upon the static nature of classifiers. With frenzied extension and expansion of biological sequences in a postgenomic era, one of the most complex and critical issues in bioinformatics is to identify the suitable way to define these sequences with vectors based on unique models. Such notations and transformations assist in maintaining the unique arrangement of sequence characteristics and essential information about proteomic data. Machine learning algorithms are incorporated to use vectors for entertaining them, but a dataset of sequences needs to decipher among classes based on data extracted by the transformation process [52]. There is a risk that a vector which is represented in a discrete structure may mislay information about sequences completely or to bypass from complete loss of information of sequences arrangement for protein, a strategy named ‘PseAAC' [53] was suggested which stands for the “Pseudo Amino Acid Composition” [54]. This strategy has been prevalently used in all fields of proteomic calculation [55–61]. This extensive and progressive use led to the formation of three existing opened access powerful and useful softwares, called “PseAAC-Builder”, “propy”, and “PseAAC-General”, for developing different methods of Chou's special PseAAC [62] where the last one is a generalization of “PseAAC” [63]. They not only include the distinctive approach for feature extraction of proteomic data but also extend to feature vectors which include, “Functional Domain” mode, “Gene Ontology” mode, and “Sequential Evolution” or “PSSM” mode. Inspired by the complementary outcome of utilizing “PseAAC” to handle the sequences of peptide or protein, the proposed strategy of “PseAAC” was continued to Pseudo K-tuple Nucleotide Composition (PseKNC) for developing and achieving different feature vectors for RNA/DNA that have confirmed very favourable as well [64–70]. Especially, recently, an advanced web server named “Pse-in-One” [71] and “Pse-in-One 2.0” [72], which is its advanced version and can be utilized in generating any required protein/peptide vector and sequences of DNA and RNA according to the requirement of the users. Here are some methodologies used for extracting the features, to identify the specific arrangements associated with the primary protein structure.

### 2.2. Position Relative Incidence Matrix (PRIM)

The first step is to transform the primary structure of protein into a matrix form for expressing the typical features of proteins. PRIM is built by utilizing the protein sequence length. With the help of a row-major strategy, protein basic structure is converted into two-dimensional from singular dimensional. We can calculate the two-dimensional matrix by the following equation if we simply take the square root of the length of the protein.

(1) $$\begin{array}{c} n=\left|\sqrt{k}\right|, \end{array}$$

Here, *n* and *k* are the two-dimensional square matrix dimension and primary sequence length, respectively. Later on, this amino acid matrix is used in the computation of PRIM through which the development of feature vector is done. The formation structure of PRIM is 20x20. The representation of two dimensional is as follows in equation (2).

(2) $$\begin{array}{c} S_{PRIM}=\left[\begin{array}{ccccc} Y_{1}⟶1 & Y_{1}⟶2 & \cdots & Y_{1}⟶j & Y_{1}⟶20\\ Y_{2}⟶1 & Y_{2}⟶2 & \cdots & Y_{2}⟶j & Y_{2}⟶20\\ \vdots & \vdots & \cdots & \vdots & \vdots \\ Y_{i}⟶1 & Y_{i}⟶2 & \cdots & Y_{i}⟶j & Y_{i}⟶20\\ \vdots & \vdots & \cdots & \vdots & \vdots \\ Y_{n}⟶1 & Y_{n}⟶2 & \cdots & Y_{n}⟶j & Y_{n}⟶20 \end{array}\right]. \end{array}$$

Here, *Y* figures out the i^th^ position residue score relative to j^th^ type amino acid. The possible values for *j* could be 0, 1, 2, 3, 4…, and so on. This 20x20 matrix can produce a total of four hundred coefficients. Statistical moments are computed for PRIM by reducing the number of coefficient elements which is 24 in the case of PRIM computation. 10 raw, Hahn, and central moments were calculated up to order three, and hence, 30 unique features were obtained.

### 2.3. Reverse Position Relative Incidence Matrix (RPRIM)

To explore concealed and complicated characteristics of an elementary sequence of the protein that has confusion with similar sequences of other protein, a matrix is used which have 400 coefficients as it contains 20x20 dimension as PRIM, known as reverse position incidence matrix.

(3) $$\begin{array}{c} S_{PRIM}=\left[\begin{array}{ccccc} Y_{1}⟶1 & Y_{1}⟶2 & \cdots & Y_{1}⟶j & Y_{1}⟶20\\ Y_{2}⟶1 & Y_{2}⟶2 & \cdots & Y_{2}⟶j & Y_{2}⟶20\\ \vdots & \vdots & \cdots & \vdots & \vdots \\ Y_{i}⟶1 & Y_{i}⟶2 & \cdots & Y_{i}⟶j & Y_{i}⟶20\\ \vdots & \vdots & \cdots & \vdots & \vdots \\ Y_{n}⟶1 & Y_{n}⟶2 & \cdots & Y_{n}⟶j & Y_{n}⟶20 \end{array}\right]. \end{array}$$

Dimensions of the matrix mentioned above are reduced. Statistical moments are calculated for RPRIM, which have 24 elements set. 10 raw, Hahn, and central moments are calculated using 2D S_RPRIM_ up till third order, 30 unique features obtained.

### 2.4. Statistical Moments

In recognition of patterns, many research methodologies demonstrate that statistical moments are fruitful to generate features against those sequences which do not rely upon any guideline. A specific category of biased average, which is used in analyzing the consolidation of some unique structure in problems related to sequence recognition is known as moments [73]. These are also helpful in many issues related to pattern recognition. Another important method for determining and understanding different kinds of sequences and object depiction is orthogonal moments.

By using techniques of polynomial and distribution functions, many statisticians develop certain moments. Further, Hahn, central, and raw moments are utilized to explain the problem in discussing in this study. There are two types of orthogonal moments, (1) discrete moments and (2) continuous moments. It has been considered in a recent study [74] that for quantized and distinct data, the result gained by a discrete moment was much better than a continuous moment. A different form of the moment can be calculated by the matrix or vector collection which represents any pattern. The raw moments are treated as generally known moments which can be calculated using the below equation (4).

(4) $$\begin{array}{c} M_{xy}=\underset{i}{\sum }\underset{j}{\sum }i^{x}j^{y}f\left(i,j\right). \end{array}$$

The origin of data is considered as a remark point by the raw moments; on the other hand, components that are far away from the origin point are used in calculating the moments. The data's centroid is used by central moments as their remark point, which was calculated by the following equation (5).

(5) $$\begin{array}{c} U_{xy}=\underset{p}{\sum }\underset{q}{\sum }\left(p-p^{\prime }\right)pow\;x\left(q-q^{\prime }\right)pow\;yf\left(p,q\right). \end{array}$$

Distinct features up to third order are obtained with the help of central moments and defined as U_00_, U_01_, U_10_, U_11_, U_02_, U_20_, U_12_, U_21_, U_30,_ and U_03_. Now, the centroids p′ and q′ are computed from equations (11) and (13).

(6) $$\begin{array}{c} p^{\prime }=\frac{\text{the }M^{10}}{M^{00}},\\ q^{\prime }=\frac{M^{01}}{M^{00}}. \end{array}$$

Orthogonal moments which need a square matrix input data in two-dimensional are Hahn moments of two dimensional. They can be calculated when the notations of one-dimension are converted into square matrix notations. N order of Hahn polynomial is calculated from the Eq. (7).

(7) $$\begin{array}{c} h_{n}^{u,v}\left(r,n\right)={\left(N+1+r\right)}_{n}{\left(N-1\right)}_{n}, \end{array}$$

(8) $$\begin{array}{c} \overset{\text{n}}{\underset{\text{k}=0}{\sum }}{\left(-1\right)}^{\text{k}}\frac{{\left(-\text{n}\right)}_{\text{k}}{\left(-\text{r}\right)}_{\text{k}}{\left(2\text{N}+\mu +\text{v}-\text{n}-1\right)}_{\text{k}}}{{\left(\text{N}+\text{v}-1\right)}_{\text{k}}{\left(\text{N}-1\right)}_{\text{k}}}*\frac{1}{\text{k}!}. \end{array}$$

Generalization of the Pochhammer symbol is made as in equation (9).

(9) $$\begin{array}{c} {\left(a\right)}_{k}=a\left(a+1\right)\cdots .\left(a+k-1\right). \end{array}$$

The Pochhammer symbol will become more simplified when using an operator named Gamma as follows in equation (17)

(10) $$\begin{array}{c} {\left(a\right)}_{k}=\frac{\Gamma \left(a+k\right)}{\Gamma \left(a\right)}. \end{array}$$

Raw values for Hahn's moments are generally measured by utilizing a square norm and weighting method, as shown in Eq. (22).

(11) $$\begin{array}{c} h_{n}^{ὐ,v}\left(r,N\right)=\sqrt{\frac{\rho \left(r\right)}{d_{n}^{2}},}n=0,1,\cdots N-1. \end{array}$$

On the other hand, in equation (12).

(12) $$\begin{array}{c} \rho \left(r\right)=\frac{\Gamma \left(r+\mu +v\right)+\Gamma \left(r+v+1\right){\left(r+1+\mu +v\right)}_{N}}{\left(v+\mu +2r+1\right)n!\left(N-r-1\right)!}. \end{array}$$

The Hahn moments which are orthogonally normalized for discrete data of two dimensional are calculated up to three orders as mentioned in equation (13).

(13) $$\begin{array}{c} H_{ij}=\overset{N-1}{\underset{q=0}{\sum }}\overset{N-1}{\underset{p=0}{\sum }}\beta_{pq}h_{i}^{ὐ,v}\left(q,N\right)h_{j}^{ὐ,v}\left(p,N\right),m,n=0,1,2\cdots N-1. \end{array}$$

For every sequence 10 raw, 10 central, and 10 Hahn moments are calculated up to third order. Features obtained by Hahn moment are represented as H_00_, H_01_, H_10_, H_11_, H_02_, H_20_, H_12_, H_21_, H_30_, and H_03_. By using the methods mentioned above, we can obtain feature vectors, after that, they are used in training and in developing a classifier.

### 2.5. Frequency Vector

In sequences, the number of the existence of amino acid is represented by frequency; a vector is figured out for frequency distribution measurement known as frequency vector.

(14) $$\begin{array}{c} \xi =\left\{\tau_{1}+\tau_{2}+\tau_{3},\cdots ,\tau_{20}\right\}. \end{array}$$

Here, in the above equation, the occurrence frequency of an amino acid i^th^ residue is denoted by *τ*_*i*_. The primary purpose of calculating this vector is to uncover and reveal the hidden sequence compositional information. A total of 20 unique features were obtained that were used with others for training purposes.

### 2.6. Accumulative Absolute Position Incidence Vector Formation (AAPIV)

The purpose of the frequency matrix is to obtain compositional information about the sequence. Still, the knowledge about the residue relative position did not get from it, for this purpose, a vector named accumulative absolute position incident is computed, which has a length of 20 elements. In this vector, the mean of all statistical values for every endemic amino acid, appearing in a primary sequence is located at their specific locations, and 20 features are obtained from it.

This vector can be denoted as *M* and represented in equation (15):

(15) $$\begin{array}{c} M=\left\{\mu_{1,}\mu_{2,}\mu_{3,}\cdots .,\mu_{20+}\right\}. \end{array}$$

For the computation of i^th^ arbitrary AAPIV's element, below mentioned equation is used.

(16) $$\begin{array}{c} \mu_{i}=\overset{n}{\underset{M=1}{\sum }}P_{M}. \end{array}$$

### 2.7. Reverse Accumulative Absolute Position Incidence Vector (RAAPIV)

RAAPIV is generated by overturning the primary sequence and producing the AAPIV from the overturn sequence. Hence, give 20 unique features. The primary purpose of developing RAAPIV is to draw out and uncover the facts and figures from the relative residue's position of the sequences. This reverse vector is represented as

(17) $$\begin{array}{c} \Lambda =\left\{\eta_{1,}\eta_{2,}\eta_{3,\cdots ,}\eta_{20}\right\}. \end{array}$$

### 2.8. Feature Fusion

After passing through all the procedures mentioned above, multiple features were fused into one vector. PRIM and RPRIM were converted into concise data by calculating moments (such as raw, central, and Hahn) and further integrated into a feature vector as well as with AAPIV and RAAPIV. This yielded 100 features. All these features helped in defining relative positions as well as absolute positions of amino acid residues. Furthermore, frequency-based features were computed through frequency vector, which elaborated the frequency of amino acids and yielded 20 features.

### 2.9. Algorithms for Classification

The third stage of the five-step rules of Chou's is elaborated in this part, which is the formation of an operational algorithm. For classification, one of the most commonly used methodologies, Random Forest (RF) has been adopted at this stage. To compare results from the random forest “Support Vector Machine” (SVM) and “Artificial Neural Network” (ANN) were also used. In research studies related to bioinformatics, methods of ensemble learnings have been practiced [74, 75] and efficient results produced by them in terms of performance. In ensemble learning techniques, the results of all several classifiers used for solving particular problems are aggregate. The two most frequently used schemes are bagging [76] and boosting [77].

Bagging the trees which are succeeding to the previous does not depend upon the preceding trees; instead, each tree is formulated independently utilizing a bootstrap sample from the data available. In the end, the prediction is determined by a simple ballot majority. Contrary to this, trees that are next in order in boosting promulgate additional value to points that were incorrectly anticipated by a former classifier. In the end, the weighted majority determines the prediction. Random forest is built by Adele Cutler and Leo Breiman [6]. A supplementary layer of randomness is an add-on to bagging. Usually, in classification trees, the partition of each node is performed by distributing a node equally between all available variables, whereas in random forest, splitting is done by selecting perfect among the available predictor's subset which was selected arbitrary were at that node. The random forest becomes a counterintuitive approach that is firmly against overfitting and performs effectively.

Random forest is an ensemble of decision trees where the training (sample) dataset is recursively partitioned into different decision trees based on the value of a parameter. It is firmly across overfitting, fast, and scalable, which enables it to give better results with an increasing number of examples.

A random forest is also known as a random decision forest because at the time of training, tasks are operated by making a multitude of decision trees, and at the time of output, the class which is the mode of all the classes used in the process or individual trees mean evaluation is given as the final result. A pictorial representation of the random forest is shown in Figure 3.

In machine learning, SVM is a supervised machine learning model. These are selective classifiers that are formally designed by a separable hyperplane. Initially, it is introduced in the 1960s and improved in the 1990s. Its working in space example can be easily understood by points. Points of each category are separated. In case the gap between an instance of different types is more massive, more comfortable to identify the cluster. So, the primary purpose of SVM is to segregate the available data in the best possible way. For this purpose, SVM kernels are used; their primary function is to add more dimensions to low dimension space. By using the kernel, an inseparable problem can be converted to a separable problem. SVM is always implemented and practiced by the kernel. Some types of the kernel are as follow: (a) linear kernel, (b) polynomial kernel, and (c) radial basis function kernel. The main advantage of SVM is that it works well in cases where the number of dimensions is greater than the number of samples. It also performs well when the space between classes is large. It does not perform well when the available data is too large or contains too much noise. SVM was used in this study just to compare results with a random forest of cross-validation, jackknife, self-consistency, and independent testing to check the effectiveness and validity of random forest. The working of SVM can be seen in Figure 4.

The processing way of the brain is adopted as a foundation for an artificial neural network. It falls in the category of supervised learning technique which utilizes backpropagation to train data. ANN is used in solving a vast dimension of the problem. It can easily discriminate nonlinear data. ANN is a framework of coupled neurons in which the next neuron input is the output of the previous one, as shown in Figure 5. A connection is known as an edge, both edge and neuron's weight help in the learning process. In ANN, outputs of the previous neuron become the input of the next neuron. The following equation represents ANN working.

(18) $$\begin{array}{c} O_{m}=f\left(\overset{h}{\underset{b=1}{\sum }}W_{bn}*f\left(\overset{i}{\underset{a=1}{\sum }}W_{ab}X_{a}\right)\right). \end{array}$$

Here in the above equation, the input is represented by *i*, the total number of output nodes and hidden layer nodes are represented by *o* and *h*, respectively. *O*_m_ denotes every m^th^ neuron output. *X*_a_ acts as an input for node *a*. The weight of edge connecting node *a* and of input layer to node *b* of the hidden layer is denoted by *W*_ab__,_ whereas the weight of connecting output layer node to node b is represented by *W*_bn_. At last, the neuron activation function is a classical sigmoid function that is denoted as *f*.

(19) $$\begin{array}{c} f\left(x\right)=\frac{1}{1+e^{-x}}. \end{array}$$

The prior formulated benchmark dataset contains positive as well as negative samples. For all collected models, a feature vector is calculated against each of them. Every feature vector consists of Hahn, raw, and central moments of the basic structure of protein for two-dimensional depiction, RPRIM along with PRIM. Furthermore, information about the position and composition is obtained in the form of the Frequency Matrix (FM). By associating all the feature vector, so each row correlates to a unique individual specimen and forms a Feature Input Matrix (FIM). Then, a matrix is acquired in an administrative aspect that adjusts to the category, i.e., negative or positive of the equivalent component in the Frequency Input Matrix. These matrices which have been discussed before, are used in training of the random forest, support vector machine and artificial neural network [75].

### 2.10. Adaptive Learning and Gradient Descent

In the training of an algorithm, gradient descent is used. This reduces the motion of the function in the contradictory route of the function's gradient and change in the rate is calculated in a further output such that

(20) $$\begin{array}{c} \theta =\theta -\gamma \nabla_{\emptyset }F\left(\theta \right), \end{array}$$

where theta *θ* is a parameter to the objective function *F*, *θ* is an element of *d*, the learning rate which is shown by *γ*, and the gradient function is represented as ∇_*θ*_*F*(*θ*). The overall algorithm efficiency depends upon the rate of learning *γ* because it ascertains the effective minimization.

There should be optimal values for the learning rate, and it is kept small, usually because more time is taken by a small percentage to join. The convergence, on the other hand, function oscillation may be caused due to the large learning rate. An adaptive learning algorithm calculates fluctuation in the learning rate and it depends on algorithm performance. On comparing the two consecutive iteration errors if an error in second as to first increases, then parameters used for that particular iteration are dismissed and the rate of learning fluctuates in a specific manner that function is downplayed by it. By usage of two consecutively calculated parameters, the weights used are again computed, and as a result, the output is also recomputed. For that ensuing run consequent errors that may occur are also calculated. Finally, on comparing with a previously calculated error rate, if it is greater than the rate of learning is diminished, furthermore, the unique rate of theta +1 is calculated and weights are eliminated as well. Likewise, the learning rate becomes high for a nominal error rate. Hence, learning rate continuously varies depending upon the execution of an algorithm.

It is observed that the learning rate can fluctuate on each point and for a parameter of each succeeding epoch these are computed as follows:

(21) $$\begin{array}{c} \theta_{n+1}=\theta_{n}-\gamma_{n}\nabla F\left(\theta_{n}\right). \end{array}$$

For the *n*^th^ epoch *γ*_*n*_ is the learning rate.

## 3. Experiment and Results

### 3.1. Prediction of Accuracy

Among many hurdles, one of the most substantial tasks in making a state-of-the-art prediction model is how the predicted model determines the rate of success objectively [58]. Focusing on this point, the proposed model requires two significant issues to examine. (1) To quantitatively express the predictor capacity and excellence, which benchmark should be used? (2) What type of test procedure is used to explore and evaluate metrics? Several parameters with different techniques for all three classifiers were used to measure the performance.

### 3.2. Test Methodology

It is essential to consider which type of test methodology should be used to examine and rate the four metrics mentioned in Eq. (2). In the examination and determination of statistics, the coming three methods are commonly utilized in the inspection and analysis of the predictor.

(1) “Subsampling” (cross-validation) test, (2) “Jackknife Test” [71], and (3) “Independent dataset test” (IDT). Out of previously mentioned testing techniques, the one which is assumed the minimum inconsistent is jackknife. Jackknife produces the slightest different output for a given dataset on testing, explained in detail in the citation [58]

In case while confirmation set is not available, for establishing an exception that the methodology that was proposed is working excellent, the cross-validation technique is used. Dataset is divided into disassociate *k*-folds in cross-validation, while *k* is preserved fixed. For each partition obtained, testing is performed *k*-times on it after computed models for every single iteration training and accuracy. In the end, the absolute accuracy mean obtained is the outcome of the subsampling testing technique cross-validation. In the current scenario to get the result, *k*-fold cross-validation has been implemented, and an arbitrary choice to generate subsets for *k* = 10 was executed.

### 3.3. Formulation of Metrics and Evaluation Parameters

Presented metrics in Eq. (23) are commonly utilized to calculate prediction's degree of excellence from four different perspectives: (a) MCC for strength and stability, (b) Acc for measuring the precision and accuracy, (c) Sp for predictor specificity, and (d) Sn for the sensitivity of the predictor [74]. Regrettably, the traditional formulation of the abovementioned was provided in [76], most experienced scientists observe difficulties in understanding them, for MCC, it is especially. Amazingly, by using Chou's letter presented in analyzing peptide signals [77] Chen et al. [6] and Xu et al. [7] transformed them into a group of four intuitive equations, which are given as follows:

(22) $$\begin{array}{c} \left\{\begin{array}{c} Sn=\frac{TP}{TP+FN}\\ \frac{Sp=TN/TN+FP}{Accuracy=TP+TN/TP+FP+FN+TN}\\ MCC=\frac{TP*TN-FP*FN}{\sqrt{\left(TP+FP\right)\left(TP+FN\right)\left(TN+\text{F}P\right)\left(TN+FN\right)}} \end{array}\right.. \end{array}$$

A symbol used for the conventional equation was introduced in ref. To define the equation, *N*_+_^−^, *N*_−_^+^, *N*^+^, and *N*^−^ symbols were used. Their details are available in Table 2.

Substitute symbols of Table 2 to Eq. (22) we get Eq. (23)

(23) $$\begin{array}{c} \begin{array}{c} Sn=1-\frac{N_{-}^{+}}{N^{+}}\\ Acc=1-\frac{N_{-}^{+}+N_{+}^{-}}{N^{+}+N^{-}}\\ Sp=1-\frac{N_{+}^{-}}{N^{-}}\\ MCC=\frac{1-\left(\left(N_{+}^{-}/N^{-}\right)+\left.N_{-}^{+}/N^{+}\right)\right.}{\sqrt{\left(1+\left.N_{-}^{+}+N_{+}^{-}/N^{-}\right)\right.\left(1+\left.N_{+}^{-}+N_{-}^{+}/N^{+}\right)\right.}} \end{array}. \end{array}$$

Eq. (21) and Eq.(20) have the same meaning but it becomes easy to understand what that equation means. Eq. (21) description is available in Table 3.

Thus, by equation (23), the overall accuracy, specificity, sensitivity, and MCC can be easily understood compared to the equation defined in (22) which is authenticated only forsingle-label systems. A real unique metric set is required for systems that are multilabelled as described in [78] and whose emergence is becoming common in biomedicine [79], system medicine [80], and system biology [81].

## 4. Discussion

Here, it is vital before going into the result section, to discuss the techniques used to get these results. As mentioned above, there are usually three popular testing techniques, (1) 10-fold cross-validation, (2) independent testing, (3) jackknife testing, and (4) self-consistency were used to validate the accuracy of the predictor model. So, in DNAPred_Prot, all the techniques were used to examine the accuracy of the proposed model. The classifier used in testing and training of the model was “Random Forest”, “Support Vector Machine”, and “Artificial Neural Network”.

The accuracy achieved by DNAPred_Prot for the prediction of DNA binding proteins is better than models [14, 40] proposed previously. DNAPred_Prot results achieved can also be viewed in graphical representation; moreover, receiver operation characteristic curves for each testing technique were also done for more precise and efficient analysis. In the end, the web server was developed using a flask framework. It was done by following the five-step rule to facilitate others with these findings.

### 4.1. 10-Fold Cross-Validation

Using a 10-fold cross-validation testing technique, an accuracy of 94.97%, 48.55%, and 79.5% was achieved with random forest, support vector machine, and artificial neural network, respectively. The results obtained from 10-fold cross-validation via random forest demonstrate that an overall accuracy obtained is highly acceptable than previously proposed predictors and SVM and ANN classifiers. Overall predicted results obtained from Eq. (23) and comparison with other existing methodologies are shown in Table 4. The ROC comparison for 10-fold, 5-fold cross-validation of random forest, artificial neural network, and support vector machine are shown in Figures 6 and 7, respectively.

### 4.2. Boxplot Visualization

Box plot is a convenient and straightforward way of displaying a set of data on scale intervals. For analysis of 10-fold cross-validation result boxplots for each classifier RF, ANN, and SVM are shown in Figure 8, Figure 9, and Figure 10, respectively.

### 4.3. Jackknife Testing

To check the quality of the predictor, we also make use of jackknife testing. In the process of jackknife testing, training and testing datasets are opened, and every sample is lifted between the two. Using this technique “Memory” effect and unforeseen problems can be removed in test and independent dataset subsampling, as from a unique dataset, always the impressive result is obtained by using jackknife testing. Results obtained in the process of recursive training via the random forest are 95.11% accurate, whereas 79.5% and 48.56% accuracy achieved by artificial neural network and support vector machine, respectively, which shows that random forest performs better than the other two classifiers. The results of all three classifiers used in this study are shown in Table 5, while ROC is shown in Figure 11.

### 4.4. Independent Testing

In independent testing, the dataset is divided into two subsamples, testing and training, first subsample training contains 70% of the dataset and the second testing subsample consists of 30%. Using the random forest technique, 97.33% accurate results were achieved which is better than 20.88% with support vector machine and 79.51% with artificial neural network, training and testing, respectively. The results of all three classifiers used in this study are shown in Table 6, while ROC is shown in Figure 12.

### 4.5. Self-Consistency

Hastie and Stuetzle in 1989 introduced the term “self-consistency” which becomes the fundamental concept in the field of statistics. It gives the suitable method for a lot of techniques in statistics which led to a more straightforward and more accessible structure for distributions representation by self-consistency, results via random forest obtained are 95.11% accurate, and 79.5% and 48.56% accuracy is obtained by support vector machine and artificial neural network which shows random forest classifier performs better. The results of all three classifiers used in this study are shown in Table 7. Also, the ROC of self-consistency for all three classifiers is shown in Figure 13.

### 4.6. Comparison with State-of-the-Art Approaches

Using the jackknife testing technique on the standard dataset for the sake of metrics represented in Equation (23), the results obtained by this methodology have an accuracy of 95.11%. To facilitate and comfort, a comparison from the different existing state-of-the-art methodologies with jackknife testing results of this methodology is shown in Table 8 and Table 9. To have a clear view and understanding of the comparison, a bar chart is also shown in Figure 14. It is visible from the table that DNAPred_Prot for metrics, i.e., accuracy, sensitivity, and MCC scores are much high. It indicates that the suggested anticipator is advanced in all four parameters on which the prediction is made for the identification of DNA-binding protein which are stability, sensitivity, specificity, and overall accuracy with its counterparts.

The comparative analysis provided in Table 9 shows that the proposed model with Random-Forest as classifier outperforms all previous existing methods and provides an accuracy of 0.914 on the independent dataset (PDB186).

### 4.7. Web server

Developing a convenient web server is the 5^th^ step in the five-step rule. As specified and explained in the number of recent publications [73–75, 81, 82], for development of practical, more useful forecasting methods and tools for computation in the future need a web server that is publicly available at the link and easy to use. The user can follow a series of steps to take benefit from the study using a web server. Steps are provided below.

*Step 1*. Open your browser and go to (https://share.streamlit.io/waqarhusain/dnapred_prot/main/app.py). It can also be seen from Figure 15 that the first page that open is the home page

*Step 2*. For prediction, input sequence in the sidebar input field. You can also find example data by clicking Example button

*Step 3*. After entering data, press SUBMIT to perform prediction. Results are shown on the main page in a tabular form. Specifically, a lot of practically important web servers have a rising impact on medical science and get it into a never known before kind of revolution. We serve our attempt for the analysis, examination, and prediction of the approach proposed in this paper by building a web server

## 5. Conclusion

DNA-binding protein plays a vital role in a lot of biological activities like transcription, DNA recombination, replication, modification, and repair. The present study is dedicated to the identification of DNA-binding protein following the five-step rules. In consideration of this intention, position relative and statistical features were integrated into DNAPred_Prot. Popular verification testing techniques jackknife and cross-validation were utilized to check the proposed model's capability and efficiency. It is crystal clear from the results that random forest performs best among support vector machines and artificial neural networks. Results of a random forest classifier using 10-fold cross-validation and jackknife's approach include 94.97% and 95.11% accurate results achieved, respectively. These results are better as compared to results obtained by support vector machine and artificial neural network. The system's overall accuracy is 95.11% to the sensitivity of 99.75% and specificity of 76.78%. It is to wind up that there is a capability in this model to be more improved in result computation as the number of protein sequences increases.

## Figures and Tables

**Figure 1:** DNA binding protein bound to respective target DNAs. Created from PDB (a) 1LMB and (b) 1 RVA. Image source [6, 7], respectively.

**Figure 2:** Flowchart of the proposed methodology.

**Figure 3:** Representation of random forest classifier.

**Figure 4:** Representation of support vector machine.

**Figure 5:** Artificial neural networks working representation.

**Figure 6:** ROC comparison for 10-fold cross-validation.

**Figure 7:** ROC comparison for 5-fold cross-validation.

**Figure 8:** Box plot for Random Forest.

**Figure 9:** Box plot representation for ANN.

**Figure 10:** Box plot representation for SVM.

**Figure 11:** ROC for jackknife testing.

**Figure 12:** ROC of independent testing by classifiers.

**Figure 13:** ROC comparison for self-consistency.

**Figure 14:** Jackknife results compared with the state-of-the-art predictors.

**Figure 15:** Visualization of the web server.

**Table 1:** Detail of the dataset used.

Sequences	Benchmark dataset	Independent dataset
Negative sequences	45,668	93
Positive sequences	11,526	93
Total	57,194	186

**Table 2:** Description of equation symbols.

Symbols	Description
*N* ^+^	The total number of true DNA-binding proteins
*N*_−_^+^	The total number of true DNA-binding proteins incorrectly predicted as nonbinding proteins
*N* ^−^	Total number of true non-DNA-binding proteins
*N*_+_^−^	The total number of true non-DNA-binding proteins incorrectly identified as DNA-binding proteins

**Table 3:** Description of possible values.

When,	Then,	Details
*N*_−_^+^ = 0	Sn = 1	None of the DNA-binding proteins is predicted as non-DNA-binding protein
*N*_−_^+^ = *N*^+^	Sn = 0	All of the DNA-binding protein is incorrectly predicted as non-DNA-binding protein
*N*_−_^+^ = 0	Sp = 1	None of the non-DNA-binding proteins is incorrectly predicted as DNA-binding protein.
*N*_+_^−^ = *N*^−^	Sp = 0	All of the non-DNA-binding proteins incorrectly predicted as DNA-binding proteins
*N*_−_^+^ + *N*_+_^−^ = 0	MCC = 1, ACC = 1	None of the DNA-binding protein and none of non-DNA-binding protein was incorrectly predicted
*N*_−_^+^ = *N*^+^and *N*_+_^−^ = *N*^−^	MCC = −1, ACC = 0	All of the DNA-binding protein and all of non-DNA-binding protein was incorrectly predicted
*N*_−_^+^ = (*N*^+^/2)and *N*_+_^−^ = *N*^−^/2	ACC = 0.5, MCC = 0	Overall prediction is not good enough than any other random prediction outcomes.

**Table 4:** 10-fold cross-validation results.

Classifier	True positive	False positive	True negative	False negative	Accuracy
Random Forest	45,480	2,748	8,778	127	94.97%
Artificial neural network	45,540	11,404	112	67	79.5%
Support vector machine	21,529	5,314	6,212	24,078	48.55%

**Table 5:** Accuracy obtained from jackknife testing.

Classifier	True positive	True negative	False positive	False negative	Accuracy
Random Forest	45,492	8850	2,676	115	95.11%
Artificial neural network	45,540	11,404	112	67	79.5%
Support vector machine	21,529	5,314	6,212	24,078	48.55%

**Table 6:** Confusion matrix obtained from independent testing.

Classifier	Type	True positive	True negative	False positive	False negative	Accuracy
Random Forest	Testing	13,693	3,044	450	7	97.33%
Support vector machine	Testing	95	3,483	11	13,551	20.88%
Artificial neural network	Testing	13,646	0	3,494	0	79.61%

**Table 7:** Accuracy obtained by self-consistency.

Classifier	True positive	True negative	False positive	False negative	Accuracy
Random Forest	45,474	8,859	2,667	133	95.1%
Artificial neural network	45,365	23	11,503	242	79.44%
Support vector machine	6212	5314	24078	21529	48.56

**Table 8:** Comparison of jackknife results with state-of-the-art predictors.

Metric/method	ACC	Sensitivity	Specificity	MCC
iDNA-Prot	0.7540	0.8381	0.6473	0.5000
PSSM-DT	0.7996	0.8191	0.7800	0.6220
DNA-binder	0.7358	0.6647	0.8036	0.4700
DNA-Prot	0.7255	0.8267	0.5976	0.4400
StackDPPred	0.8996	0.9112	0.8880	0.7990
DNAPred_Prot	**0.9511**	**0.9975**	**0.7678**	**0.8444**

**Table 9:** Comparison of independent dataset PDB186 on the proposed method with other predictors.

Method	ACC	Sensitivity	Specificity	MCC
PSSM-DT	0.8000	0.8709	0.7283	0.6470
iDNA-Prot	0.6720	0.6770	0.6670	0.8330
DNA-Prot	0.6180	0.6990	0.5380	0.2400
DNAbinder	0.6080	0.6990	0.5380	0.2400
DNA-BIND	0.6770	0.6670	0.6880	0.3550
DBPPred	0.7690	0.7960	0.7420	0.5380
StackDPPred	0.8655	0.9247	0.8064	0.7363
KKDBP	0.8120	0.9780	0.6450	0.6610
MKSVM (with MKL-CKA)	0.8370	0.9360	0.7420	0.6910
MK-FSVM-SVDD	0.8550	0.9570	0.7530	0.7250
FTWSVM-SR	0.8660	0.9460	0.7850	0.7410
TWSVM	0.8330	0.9460	0.7200	0.6840
DBP-PSSM	0.8118	—	—	0.657
DNAPred_Prot (proposed)	**0.9140**	**0.9785**	**0.8495**	**0.8349**

## Data Availability

The data are available through online server: https://share.streamlit.io/waqarhusain/dnapred_prot/main/app.py.
